This article has been retracted.

# Innovative Research on Urban Community Governance Decision-Making Relying on Distributed High-Performance Computing Blockchain Key Algorithms

**DOI:** 10.1155/2022/4078014

**Published:** 2022-03-15

**Authors:** Jun Wen, Peihong Xie

**Affiliations:** ^1^School of Cultural Creative Industries Management, Shanghai Institute of Visual Arts, Shanghai 201620, China; ^2^School of Management, Shanghai University of International Business and Economics, Shanghai 201620, China

## Abstract

Since the country began to go global, the country's economy has developed rapidly, cultural exchanges between countries have become more and more frequent, and foreign cultures have begun to gradually spread to the country. At the same time, through the absorption of foreign community governance experience, domestic research on community governance has also begun to be put on the agenda. This paper aims to study the innovative exploration of urban community governance mechanisms through key high-performance computing algorithms. To this end, this paper proposes a combination of the Bayesian algorithm and distributed high-performance computing to analyze and explore the governance and management methods of the community through its efficient and stable computing power, and derive the most suitable community governance mechanism. An experiment was also set up for comparative analysis. The experimental results show that the community governance mechanism derived from the key distributed high-performance computing algorithm improves the community governance capability by 19.4%, effectively improving the community governance and management issues.

## 1. Introduction

In recent years, with the rapid development of Chinese politics, economy, and society, the process of urbanization has accelerated, and residential privatization has continued to advance. In a sense, Chinese cities are divided into multiple functional communities. Community is the basic unit of social management and bears the responsibility of building a harmonious society. At the beginning of 2010, the outline of China's national economic and social development's 12-year plan proposed to fully implement the construction of urban communities, improve the new type of community management and service system, and build communities. It promotes the urbanization process of community construction, expands the management model, improves the service management system, accelerates the pace of marketization and modernization, and builds a harmonious socialist society.

The themes of construction, development, and governance of urban communities have received more and more praise from political parties, experts at all levels, scholars, and urban residents. Moreover, with the further development of urban community construction, the diversity governance of urban communities has also produced huge social benefits. Urban community governance is an important foundation of urban governance in the new era, the basic work of modern city construction, and an important part of the reform of modern city management systems. According to specific conventions, it is recommended to build an urban community governance mechanism. By strengthening the construction of adjusted governance mechanisms such as participation in decision-making, response governance, and public consultation, the opposition in urban community governance in the policy system will be fundamentally resolved and alleviated. In order to comprehensively improve the efficiency of urban community governance, it is necessary to promote the improvement of Chinese urban governance system and the modernization of governance capabilities. Through the use of distributed computing and key blockchain algorithms, it is very necessary to govern urban communities.

The research on the construction of foreign cities is relatively mature compared with China. Research uses the path from practice to theory, and then applies theory to practice. The research results mainly focus on the impact of social changes in urban communities, the research on the operating mechanism and process of urban communities, and the types of urban communities. A new parallel approximate Bayesian computational sequential Monte Carlo (pABC SMC) algorithm proposed by Jagiella et al. allows robust data-driven modeling of multi-scale biological systems, and proves the feasibility of multi-scale model parameterization through statistical inference [1]. However, the algorithm is mainly based on the parameters obtained by inference on the theoretical basis, and has not been verified by the experimental area. The interactive high-performance computing proposed by Mundani et al. is undoubtedly beneficial to many computing science and engineering applications, as long as the simulation results be visualized in real time during the calculation process. Because a few gigabytes of data per second is not uncommon for running simulations, a new method based on the sliding window technology is introduced and allows users to interactively study the large-scale and small-scale effects of the simulation results [2]. The problem of real-time visualization processing in the calculation process has not been solved well. JUDEHOWELL has studied the process of adaptive governance and authoritarian resilience from the perspective of community governance, bringing together unrelated research fields so far. He believes that adaptation will have unintended consequences and may threaten stability, but it will not necessarily lead to a political crisis [3]. Mullen has spent decades developing tools for the High-Performance Computing (HPC) community, teaching practitioners to use the power of parallel and distributed computing to familiarize student users with their target systems. The course materials are presented through the lens of common HPC use cases and parallelization strategies so that students are able to achieve performance improvements on their HPC systems [4]. However, the learning path of the students is still not clear enough, and the relevant display is not enough. Palmer B introduced the GridPACK™ framework, which is designed to help grid engineers develop modeling software that can run on high-performance computers. GridPACK™ contains modules for setting up a distributed grid network, assigning buses and branches with arbitrary behavior to the network, creating distributed matrices and vectors, and using parallel linear and nonlinear solvers to solve algebraic equations [5]. But there is no clear introduction to how the framework works on related modeling software. The problem of Turek simulating micro-scale urban traffic in a large environment provides a huge opportunity for the use of HPC systems. The parallel implementation of this calculation is not simple. The simulation proposed in his article is based on the concept of controlled desynchronization of computation, which does not violate the model. The implementation of the Erlang language uses the Erlang distribution mechanism to build and manage computing clusters [6]. The difficulty in the parallel realization of the calculation process is still lack of explanation, which leads to the lack of clear understanding of the HPC system. Alawneh L believes that if you use trace analysis, you can more easily understand the interaction between the processes of the high-performance computing (HPC) system. So, he proposed a novel tracking abstraction method designed to facilitate the analysis of large-scale execution tracking generated by HPC applications. Their method allows the automatic segmentation of large traces into smaller and meaningful clusters, which reflect the various execution stages of the trace scenario [7, 8]. But there is no good elaboration on the principle of this novel tracking abstract method. The purpose of Arya and Wijaya's research is to let people know more about the role of women on the coast of Surabau. The role of coastal women is not limited to their family role, and through social capital management, coastal women can also contribute to local governance. Research has found that coastal women groups can achieve success in social bonds, bridges, and connections. Under the leadership of a sufficiently effective women's group to manage the organization, people realized the need for a savings movement and had a process of sharing information and knowledge. The social bridge capital shown for establishing connections with other groups also provides a foundation for the construction of an urban society from another angle, which is convenient for later development [9]. The above documents are still very detailed for their main technologies, and the research on some technologies is also very in-depth. However, the above-mentioned literature mainly studies the related application fields of high-performance computing, and the research on its actual operability is not enough, and it is easy to have problems in the actual use process.

The innovation of this paper is to use the key algorithm extraction of the blockchain combined with distributed high-performance computing as the technical support, the urban community governance theory as the theoretical support, and the research and analysis of the urban community governance as the research object. And in the experiment and analysis part, related experiments are designed to explore the effect of its governance, to ensure that the improved governance mechanism can be effectively implemented in practice. In addition, two key algorithms were selected for comparative analysis. On this basis, some more mature urban community governance theories in foreign countries were used to construct a governance path, learn from its experience, select the essence, and remove the dross, which combines the governance methods of China's socialist society to deduct the governance of urban communities, and with the support of high-performance computing capabilities, it deduces a governance method that is more suitable for most communities and improves the governance mechanism of the community.

## 2. High-Performance Computing Methods

### 2.1. Blockchain Cloud Computing Method

Cloud computing is a paid service, and users need to purchase corresponding cloud computing services on demand under the premise of fully evaluating their own situation. Cloud computing implements the abstraction of resources such as data computing, data storage, network transmission, and hardware equipment through key technologies such as virtualization, distributed parallel processing, and the Internet, and then provides these resources to users dynamically on demand. This provides users with a more flexible, convenient, and economical way to dynamically obtain computing resources and storage resources according to their needs [10]. For users, instead of purchasing and maintaining huge and expensive infrastructure and incurring huge costs, it is obviously better to dynamically and expandably rent the necessary cloud computing resources and storage resources according to their needs. In this way, users can not only avoid early-stage investment risks, but also avoid the inability of resources to meet demand due to the increase in the company's scale, which is very attractive to small- and medium-sized enterprises, especially start-ups. Although cloud computing is considered to be the service model of the next generation Internet and cloud computing services have become more and more perfect after this year's rapid development and research, data security and privacy protection are still the main challenges that currently restrict the further development of the cloud computing field (location information protection, mobile phone data protection, authority protection, etc.). Unlike the traditional computing model where users fully control data calculation and storage locally, cloud computing requires the user's data and physical servers to be centrally managed by the cloud service provider, and the user only retains some control rights over the leased virtual machine [11], The advantages of traditional computing models compared with cloud computing models are mainly focused on the security protection of data because they completely control local data and storage, thus having higher security. The cloud computing method application service of blockchain is shown in Figure 1:

There are three common deployment models for cloud computing: public cloud, private cloud, and hybrid cloud. Users can choose to use different deployment models according to the type of data to be processed and the requirements for security and data management [12].

Public Cloud: In the public cloud, service providers use the Internet to provide users with computing resources including applications and storage. Public clouds are operated by third-party providers, and applications and service requests from different users are collectively run and processed on cloud servers, storage systems, and networks. Public cloud has the advantages of low cost, no maintenance, high scalability, and high reliability [13].

Private Cloud: A private cloud is a cloud computing service dedicated to a single user, which can be regarded as a user's private data service center. In a private cloud, infrastructure and services are managed and maintained on a dedicated network, and software and hardware services only serve a single user. Private clouds can also be operated and maintained by third-party service providers. Private clouds are often favored by users who are sensitive to data security, such as government agencies and financial institutions. Private cloud services have the advantages of more flexibility, higher security and reliability, and high open scalability.

Hybrid Cloud: Hybrid cloud combines the user's infrastructure or private cloud and public cloud to obtain the advantages of both at the same time. In a hybrid cloud, data and applications can be securely transferred between private and public clouds for greater flexibility and more deployment options. Users can use the public cloud to perform operations with high storage capacity and low security while using the private cloud to perform secure operations on sensitive businesses. Hybrid cloud combines the advantages of the previous two, with advantages such as controllability and flexibility.

Cloud computing implements the abstraction of data computing, data storage, network transmission, and hardware equipment through key technologies such as resource management, distributed parallel processing, and the Internet, and then provides these resources to users dynamically on demand. Taking into account the above characteristics, this article adopts the hybrid cloud deployment model for related deployment. This service process mainly involves three aspects of technology, including resource management, Internet technology, and distributed computing. The research on distributed computing is the focus of this article. As shown in Figure 2, it is the key technology involved in the cloud computing process [14].

Resource management technology mainly includes virtualization technology and data center management technology. Virtualization technology is one of the core key technologies of cloud computing, which can abstract the details of physical hardware and provide virtualized resources for advanced applications. Virtual machine services with scalable performance can be provided to users through virtualization technology, which further improves the utilization efficiency and high scalability of physical servers in the case of multiple users. Data center is the core of the cloud computing architecture. Data center management technology is one of the most basic core technologies of cloud computing, which directly affects the performance of upper cloud data storage and computing services. Cloud computing data centers include technologies such as network topology, large-scale data storage, resource management and scheduling, and they need to have features such as autonomy, economies of scale, and scalability. In cloud computing, Internet technology is used to complete the interaction between the users and cloud resources. Cloud computing only requires the user's data and physical servers to be centrally managed by the cloud service provider, and the user only retains some control over the leased virtual machine. At present, most cloud computing service providers provide users with web-based cloud interactive interfaces. The B/S architecture-based approach not only reduces the development cycle, but also further reduces the resource occupation of the client [15].

### 2.2. SVM Algorithm Optimization for Distributed Computing

#### 2.2.1. Classification of Classification Algorithms

*(1) Decision Tree Algorithm*. The decision tree method is to first find the most informative attributes in the sample database as the nodes of the decision tree, and then construct various branches of the nodes according to the attribute values. Then, repeat this process for each one. It is used to establish the branch of the next node and its branches [16].

*(2) Bayesian Classification*. Bayesian classification is a statistical classification method. The classification principle is to use the pre-probability of the object and use the Bayesian equation to calculate the post-probability. In other words, the object has the probability of belonging to a specific category, and the category with the largest posterior probability is selected as the class the object belongs to [17].

For a training sample, suppose its prior probability is *P*; according to Bayesian classification, the probability obtained is

(1) $$\begin{array}{c} p\left(z\right)=p\left(z/si\right)\cdot p\left(si\right)/p\left(x\right). \end{array}$$

If

(2) $$\begin{array}{c} p\left(si/z\right)=\text{Max}jp\left(sj/Z\right),i=1,2,3\cdots ,N, \end{array}$$

then there is *x* ∈ *si*; substituting formula (1) into formula (2),

(3) $$\begin{array}{c} p\left(z/si\right)p\left(si\right)=\text{Max}j\left[p\left(z/sj\right)p\left(sj\right)\right],i=1,2,3,\cdots N,j=1,2,\cdots ,N. \end{array}$$

This is the most commonly used Bayes classification decision benchmark. As a result of years of research, the Bayesian classification is widely used. However, because the Bayesian sample size is large enough, the sample properties must be independent of each other; it is difficult to achieve this in practical applications, and hence it is difficult to achieve theoretical results with this method [18].

*(3) Neural Network Classification*. As shown in Figure 3, the neural network classification is mainly composed of three layers to form a multilayer feedforward neural network (Input layer, hidden layer, output layer) [19]. The multilayer feedforward neural network consists of an input layer, one or more hidden layers, and an output layer. The Back Propagation [BP] algorithm learns on the multilayer feedforward neural network, and the [multilayer] feedforward neural network using the BP algorithm is called the BP neural network.

The most commonly used multilayer feedforward neural network lies in classification. By setting the number of sample attribute values and controlling the sample type of the output layer, various classifications can be performed. But the problem that it is easier to fall into the minimum is one of its inherent shortcomings.

*(4) Linear Classification*. The learning goal of a linear classifier is to find a classification hyperplane in the n-dimensional data space, and its equation can be expressed as

(4) $$\begin{array}{c} \omega^{T}z+b=0. \end{array}$$

As shown in Figure 4, in the two-dimensional plane, the solid line is the classification plane. We can make the classification function as

(5) $$\begin{array}{c} f\left(Z\right)=\omega^{T}z+b. \end{array}$$

At the same time, use *z* to represent the “geometric distance” of the classification hyperplane;

(6) $$\begin{array}{c} \gamma =y\frac{\omega^{T}z+b}{\left|\left|\omega \right|\right|}=y\frac{f\left(z\right)}{\left|\left|\omega \right|\right|}. \end{array}$$

Its mathematical expression is as follows:

(7) $$\begin{array}{c} \underset{\omega ,b}{\min}\frac{1}{\left|\left|\omega \right|\right|},s,t,y_{i}\left(\omega^{T}z_{i}+b\right)\geq 1,i=1,2,\cdots ,n. \end{array}$$

The above problems can be equivalently transformed into the following problems:

(8) $$\begin{array}{c} \underset{\omega ,b}{\min}\frac{1}{2}{\left|\left|\omega \right|\right|}^{2},s,t,y_{i}\left(\omega^{T}z_{i}+b\right)\geq 1,i=1,2,\cdots ,n. \end{array}$$

The constraints are integrated into the objective function through the Lagrangian function, as follows:

(9) $$\begin{array}{c} L\left(\omega ,b,a\right)=\frac{1}{2}{\left|\left|\omega \right|\right|}^{2}-\sum_{i=1}^{n}\alpha_{i}\left(y_{i}\left(\omega^{T}x_{i}+b\right)-1\right). \end{array}$$

Then make

(10) $$\begin{array}{c} \beta \left(\omega \right)=\underset{a_{i\geq 0}}{\max}L\left(\omega ,b,a\right). \end{array}$$

Our question is transformed into a request:

(11) $$\begin{array}{c} \underset{\omega ,b}{\min}\beta \left(\omega \right)=\underset{\omega ,b}{\min}\underset{a_{i}\geq 0}{\max}L\left(\omega ,b,a\right). \end{array}$$

Further transformed into

(12) $$\begin{array}{c} \underset{a_{i}\geq 0}{\max}\underset{\omega ,b}{\min}L\left(\omega ,b,a\right). \end{array}$$

In order to solve equation (12), we first find the minimum values of *ω* and *b* in equation (9), and calculate the extreme values of *ω* and *b*, respectively, according to the extreme value conditions, namely:

(13) $$\begin{array}{c} \nabla_{\omega }L\left(\omega ,b,a\right)=0\\ \nabla_{b}L\left(\omega ,b,a\right)=0. \end{array}$$

Solve to get

(14) $$\begin{array}{c} \omega =\sum_{i=1}^{x}\beta_{i}\alpha_{i}y_{i}. \end{array}$$

(15) $$\begin{array}{c} \sum_{i=1}^{n}\alpha_{i}y_{i}=0. \end{array}$$

Substituting (14) and (15) into (12), the dual form of the original problem is obtained as follows:

(16) $$\begin{array}{c} \begin{array}{cc} \max\overset{n}{\underset{i=1}{\sum }}\alpha_{i} & -\frac{1}{2}\overset{n}{\underset{i,j=1}{\sum }}\alpha_{i}\alpha_{j}y_{i}y_{j} \end{array}\\ t,s,a_{i}\geq 0,i=1,2,\cdots ,n,\overset{n}{\underset{i=1}{\sum }}a_{i}y_{i}=0. \end{array}$$

That is, the original nonlinear data are mapped to a new feature space through a nonlinearity, and the following function is obtained:

(17) $$\begin{array}{c} f\left(Z\right)=\sum_{i=1}^{n}\omega_{i}\varphi_{i}\left(Z\right)+b. \end{array}$$

Assuming that the data can be obtained by the linear combination of training points, it can be expressed as the following formula:

(18) $$\begin{array}{c} f\left(Z\right)=\sum_{i=1}^{n}\alpha_{i}y_{i}<\varphi \left(Z_{i}\right)\cdot \varphi \left(Z\right)>+b. \end{array}$$

Assuming that the kernel is a function *K*, for all *x*, z ∈ *x*, satisfy

(19) $$\begin{array}{c} K\left(X,Z\right)=<\varphi \left(x\right)\cdot \varphi \left(z\right)>. \end{array}$$

Then, Φ is the mapping from *X* to the inner product feature space *F*. The Gaussian kernel *K* is

(20) $$\begin{array}{c} K\left(z_{i},z_{j}\right)=\exp\left(-\frac{{\left|\left|z_{i}-z_{j}\right|\right|}^{2}}{2\sigma^{2}}\right). \end{array}$$

That is, for any Φ(*x*) ≠ 0, there is

(21) $$\begin{array}{c} f\Phi^{2}\left(X\right)dx\;<\infty . \end{array}$$

Then, there are

(22) $$\begin{array}{c} \int \int K\left(z,z^{\prime }\right)\Phi \left(z^{\prime }\right)\text{d}z\text{d}z^{\prime }>0. \end{array}$$

We turn the linear inseparable problem into

(23) $$\begin{array}{c} \underset{a}{\max}\sum_{i=1}^{n}a_{i}-\frac{1}{2}\sum_{i,j=1}^{n}a_{i}a_{j}y_{i}y_{j}K\left(x_{i},x_{j}\right)\\ t,s,a_{i}\geq 0,i=1,2,\cdots ,n,\sum_{i=1}^{n}a_{i}y_{i}=0. \end{array}$$

By solving it, we can get an optimal SVM algorithm optimization method so as to improve it.

### 2.3. Distributed Collaborative High-Performance Computing

The collaborative computing of the distributed model refers to the realization of simulation applications by coordinating and collaborating in a distributed environment with the help of computer, network technology, and model resources. This service sharing-based model not only enables the model to run in the best operating environment and ensures the safety of the model code, but also uses more computing resources and storage space to complete various complex application simulations. Using more computing resources and storage space to complete various complex application simulations can better protect the simulated data. Therefore, DCHF-SI needs to provide a collaborative environment for remote coupling and interaction of physical models located in different locations. The interaction process of the model is transparent to the user and needs to meet the particularity of different spatial physical applications and general commercial applications; the structure of DCHF-SI is shown in Figure 5.

#### 2.3.1. Coupling Interaction Basic Framework Layer

The coupling interaction mechanism is responsible for the interaction coupling and communication of remote model components. The coupled interaction basic framework is the core supporting platform of the entire framework operation [20].

#### 2.3.2. Framework Service Component Layer

Fault-tolerant service components provide checkpoints for setting up network or grid resources and rollback recovery and other fault tolerance strategies and log strategies [21].

#### 2.3.3. Physical Model Component Layer

The physical model components are mainly obtained by encapsulating the physical model.

#### 2.3.4. Graphical User Interface (GUI) Layer

Model sharing provides researchers with a large amount of model resources. However, it is very difficult for researchers to select the model they need from the massive model resources, and it is impossible to study and analyze all the available models. In order to solve this problem, the screening of related resource models is essential. As shown in Figure 6, when the model component is coupled with the internal model, there are *M∗N* assembly methods, which makes the application assembly more complicated [22].

Therefore, this paper proposes a new type of component-abstract domain component. Models in the same domain share an abstract domain component. It also has a unified standard port for this type of model, but it is not responsible for its implementation; instead, the best model components are selected through the QOS service to participate in the calculation, thereby achieving transparent and intelligent assembly of applications and reducing the burden on developers. The following interfaces need to be added to realize the generation and connection of abstract components [23]. The design scheme of the QOS service customizable northbound interface describes the external form and the internal function model of the interface, and based on this scheme, a northbound interface that provides bandwidth and priority customizable services is implemented. The interface is tested in the SDN experimental network, and the test results show that the scheme can achieve the expected goal.

## 3. Investigation and Experiment on the Status Quo of Urban Communities

A city is a product formed to adapt to the times, a manifestation of mature economic development, and a settlement formed by a multifaceted population. As the center of trade, it continues to attract foreigners, the number of permanent residents also increases, and coupled with resource constraints and unreasonable urban layout, it has been greatly affected. In order to improve this situation, government departments have established urban communities. The specific implementation steps are: first, delineate a range, and then build concentration camps in this area, such as commercial housing communities, office communities, etc., to guide relevant people to reside in them, to save resources as much as possible, use limited space to house more people, and let them form a society with a large number of people and a high concentration of people. Housing in the city community is mostly engaged with nonagricultural work, which can accommodate people from various places and various types of work, and the rational use of space to create a small, densely populated social group. However, compared with rural areas, there is a lack of interpersonal communication [24].

At present, China's urban community governance has made great progress in terms of systems and mechanisms, but there are still many problems. There are many reasons for these problems, including the inertial effect of the original system, the influence of cultural traditions, and the lag in social development. For these issues cannot be ignored, it is necessary to explore the outstanding performance in different practices. This chapter is based on the status quo of community governance in urban communities, through combing the status of community governance practices, and discovering some potential problems in urban community governance so as to obtain beneficial enlightenment and help improve urban community governance. Here, we make a rough statistics of the number of communities within the scope of the survey statistics, as shown in Table 1:

It can be seen from the statistical data in the above table that social organizations have grown rapidly in the past two years, and the number of private units has grown relatively slowly; while foundations have no growth opportunities, the rapid growth of social organizations will lead to a management problem. If there is no good management and governance method, it is easy to cause problems. Therefore, a survey of satisfaction with the governance methods of urban community groups is added, as shown in Table 2:

Obviously, it can be seen that the problem caused by the excessively rapid growth of social organizations is that there are many governance problems, governance chaos, and the satisfaction of group members is low, while private units basically grow slowly, showing satisfaction and dissatisfaction, and the satisfactory conditions are basically the same. The foundation has grown by one in three years, and this has resulted in them having enough time to administer the foundation, so that the vast majority of people can be satisfied, and the satisfaction will naturally increase [25].

### 3.1. Weak Community Social Organizations

In the context of modern development, urban community governance, such as the introduction of the participation of social forces, can add new vitality to community services. Social organizations participating in community governance can give full play to their role as a link, integrate their own resource advantages, broaden funding sources for community governance, assume part of the governance capacity, and use their professional capabilities to provide residents with market-oriented services.

A social survey experiment on the degree of understanding of community social organizations was organized here, and the experimental data obtained are shown in Table 3:

From the above table, we can see that in urban communities, children's understanding of community social organizations accounted for 2%, adults accounted for 8%, and the elderly 2%. It only accounts for 12% of the total, and the number of people who understand it is really too small. Children and the elderly have less knowledge of community social organizations, and it is mainly concentrated that adults have more knowledge of urban community organizations. As a result, most people have problems with the governance of the community. This also reflects the problems of small-scale social organizations, insufficient development, and insufficient influence in Chinese cities. Community funding is not guaranteed, and it is easy to be administrated. The inability to independently assume the responsibility of community management has led to inadequate governance in the community [26].

### 3.2. Residents Lack Awareness of Active Participation

Serving community residents is the purpose and goal of community governance, and all governance actions are based on safeguarding the interests of the residents. The extent of residents' participation in community autonomy to a large extent reflects the true level of community autonomy. From the survey of urban community residents participating in community activities in Table 4, it can be seen that the basis for the formation of this sense of identity and belonging is gradually disintegrating [27].

Analyzing the data in Table 4, we can see that the proportion of children who often participate is 4%, adults 6%, and the elderly 2%. These values are far lower than those of a healthy and qualified urban community. The proportion of participants is only 12%, the proportion of those who have participated in some is 30%, the proportion of those who have participated occasionally is 33%, and the proportion of those who have never participated is 25%. Similarly, some seldom participate in community activities, indicating that there are fewer feedbacks on problems in this community, and people cannot conduct a good and effective management of the urban community. For this reason, we have also made a detailed survey on the reasons why people of different ages do not participate in community activities. The survey data are shown in Table 5:

From Table 5, we can still see that adults still pay attention to the interests of the majority, and this is one of the reasons why most people do not participate in community activities. The reason for this phenomenon is that the community's publicity is still insufficient, thus failing to make people develop the concept that community governance is related to everyone. This has also caused more and more people to lose confidence in community management.

Another questionnaire is designed here to investigate and reform the community governance system. There are 21 questions in the questionnaire, which consist of two parts: the first part is the basic information of the interviewee, covering nine aspects including gender, age, marital status, location of household registration, education level, residence time, identity, political outlook, and average monthly income. It forms a characterization description of the interviewee; the second part is a survey of the current community governance system. Questions include community party organizations, community neighborhood committees, community service stations, community intermediary organizations, residents' participation, community-related policies, and other elements of the community governance system.

## 4. Status Quo and Improvement of the Community

### 4.1. Relevant Situation of the Community Governance System

From the selection of residents, it can be found that almost ordinary people regard the community committee as the first choice to help them solve the difficulties in daily life, which shows that the community committee has a relatively high sense of identity in the hearts of residents, followed by government departments and community service stations. Compared with the other three governance bodies, the owners' committee and the property company do not seem to be “rooted”(the other three governance entities mainly include: private units, foundations, and social groups), which also reflects the absence of the two in community governance, which is not conducive to building a “social coordination” community governance system in the long run. The relevant situation investigation is shown in Figure 7:

From the table above, we can see that in urban communities, the number of residents who often live with neighborhood committees accounts for about 15%. Among them, children and the elderly account for more, while adults still account for a minority. About 40% of the people who don't care about the governance and management of the community and occasionally contact the neighborhood committee account for about 40%. Among them, children and adults account for a relatively large number, while the elderly are relatively small. Among those who almost never contact the neighborhood committee, adults account for the overwhelming majority, while children and the elderly account for only a small proportion. In the statistics of familiarity, the proportion of people who know the neighborhood committee is about 25%. On the contrary, the proportion of children is the largest, while the proportion of adults and the elderly is relatively small. Among those who do not know the director of the neighborhood committee at all, children and adults account for a larger proportion, while the elderly are fewer. Among those who have heard of it but are not clear, there are more adults and fewer elderly and children. The statistics on the familiarity of community party organizations and the degree of recognition of their related governance methods are shown in Figure 8:

From the survey statistics in Figure 9 on the familiarity of community party organizations and the recognition of related governance methods, we can see that the managerial personnel in the community neighborhood committees still have a relatively high percentage of recognition of the governance methods of urban communities, reaching 15.9%; in addition, the managers of all organizations have a high degree of recognition of the governance methods, and the members of them generally do not agree with the governance methods, and they are maintained at a low level. The senior citizens who agree with party secretaries are the elderly, and most adults don't know the secretaries of the community's party organizations. When the main personnel in an urban community do not know the secretaries of the community's party organization, it can only indicate the urban community. The publicity of the community is still not in place, resulting in an insufficient sense of participation of community members and the inability to actively participate in the comprehensive governance and control of the community.

In summary, the “two committees” of the community are not closely connected to the residents, and the community party organizations and community neighborhood committees are precisely the “top people” who drive residents to actively participate in community governance. Therefore, the construction of the “two committees” in the community governance system needs to be further improved and strengthened. At the same time, the problem activities organized by the community are counted, as shown in Figure 9:

From the urban community's participation in community activities organized by the community, we can see that most of the adults in cultural and sports activities have not participated in any of the activities. The main reason is to let their children participate in some activities organized by the community, but if it's just like this, it means that they have not participated in community team activities at all. Children's participation in community activities does not have much effect on the progress of the community. Similarly, in terms of public welfare activities, the majority of children participate in activities, followed by the elderly who stay at home, and most adults do not participate in the governance of the community, which reflects the fact that the activities of the community mainly remain at the level of formality, and there is no in-depth understanding of the meaning of community activities.

From the above data results, we can find that most residents are not very active in participating in community activities, and community activities are one of the effective ways to increase the sense of belonging and identity of community residents to the community. Therefore, how to improve the community governance system and eliminate the gap in public participation is worthy of our deep consideration.

### 4.2. Distributed High-Performance Computing Capability

Analyze the phenomenon in the process of urban governance through the calculation and analysis of the surveyed data, and analyze the problems of urban community governance. Therefore, it is possible to deduce a most suitable governance method, cooperate with community managers to better manage the community, and creatively explore the most suitable governance methods for each urban community.

Here, we combine the experimental data investigated by the above analysis and analyze the community governance issues through distributed high-performance computing, coordinate the role of various organizations in urban communities, and actively guide community members to participate in the governance of the community. The analysis data are shown in Figure 10:

From the above Figure 10, we can see that the development distribution curve of the community is more concentrated, which is more conducive to the stable construction of the urban community. Regarding the exponential growth of the community, the environment of the urban community has increased by 21.1% compared with previous years, and the community is safer than in previous years. With an increase of 11.1%, the development of urban communities has increased by 26% compared to previous years. The overall situation shows growth; it can be seen that using distributed high-performance computing to calculate the various factors of the community, the most suitable community development plan can be deduced, which is more conducive to the development of the community. After implementation, the overall urban community governance has increased by 19.4%.

The data obtained through calculation and analysis is more conducive to our assumption of a sound and harmonious urban community and the establishment of a democratic rule of law, fairness and justice, honesty and friendship, full of activities, stability and order, and harmonious coexistence between people's living environments.

## 5. Conclusions

This paper mainly conducts innovative research on the current domestic urban community governance methods, mainly using the computing power of distributed algorithms and the use of key algorithms of blockchain technology, and comprehensively analyzes and understands the current community through the combined use of the two. The goal of improving the current domestic community management dilemma has been achieved by exploring the management methods and improving the management methods. At the same time, the analysis and comparison of the urban community governance mechanism after the analysis of distributed high-performance computing is carried out, and it is found that through the calculation derivation the proposed governance method can improve the overall governance effect of the community by 19.4%. It can be seen that the use of related distributed algorithms in this paper is effective, and the improved management method can promote the development of the community toward a stable and harmonious direction.

## Figures and Tables

**Figure 1:** Application services of blockchain cloud computing.

**Figure 2:** Key technologies involved in cloud computing.

**Figure 3:** Multilayer feedforward neural network.

**Figure 4:** An example graph of 2-dimensional separability.

**Figure 5:** DCHF-SI structure diagram.

**Figure 6:** Model component and internal model component coupling description.

**Figure 7:** Statistics on the frequency and familiarity of residents' contact with neighborhood committees.

**Figure 8:** Statistics on the familiarity of community party organizations and the degree of recognition of their related governance methods.

**Figure 9:** Residents' participation in cultural and sports activities and public welfare activities organized by the community.

**Figure 10:** The distribution curve of urban community development and the exponential growth of all aspects of the community.

**Table 1:** Statistics on the number of urban community groups.

Group	Social groups	Private unit	Foundation
2016	75	32	9
2017	91	38	9
2018	114	43	10

**Table 2:** Satisfaction of urban community groups.

Group	Social groups	Private unit	Foundation
Satisfy	56	221	389
Dissatisfied	489	243	31

**Table 3:** Urban community residents' understanding of community social organizations.

Generation	Very familiar (%)	Probably understand a little (%)	Don't understand at all (%)
Child	2	8	18
Adult	8	31	2
The elderly	2	10	17

**Table 4:** Urban community residents' participation in community activities.

Condition	Child (%)	Adult (%)	The elderly (%)
Often attend	4	6	2
Participated in some	10	17	3
Participate occasionally	8	20	5
Never participated	7	15	3

**Table 5:** Participation in community activities by people of different ages.

Condition	Child (%)	Adult (%)	The elderly (%)
No benefit	1	30	4
No time to	2	12	3
No effect	3	15	5
Don't know to Participate	8	1	3
Never heard of that	6	3	4

## Data Availability

The data used to support the findings of this study are available from the corresponding author upon request.

## References

[1] Jagiella N., Rickert D., Theis F. J., Hasenauer J. (2017). Parallelization and high-performance computing enables automated statistical inference of multi-scale models. *Cell Systems*.

[2] Mundani R. P., Frisch J., Varduhn V., Rank E. (2018). A sliding window technique for interactive high-performance computing scenarios. *Advances in Engineering Software*.

[3] HOWELL J. (2016). Adaptation under scrutiny: peering through the lens of community governance in China[J]. *Journal of Social Policy*.

[4] Mullen J., Byun C., Gadepally V., Samsi S., Reuther A., Kepner J. (2017). Learning by doing, high performance computing education in the MOOC. *Journal of Parallel and Distributed Computing*.

[5] Palmer B., Perkins W., Chen Y. (2016). GridPACK: a framework for developing power grid simulations on high performance computing platforms. *International Journal of High Performance Computing Applications*.

[6] Turek W. . (2017). Erlang-based desynchronized urban traffic simulation for high-performance computing systems. *Future Generation Computer Systems*.

[7] Alawneh L., Hamou-Lhadj A., Hassine J. (2016). Segmenting large traces of inter-process communication with a focus on high performance computing systems. *Journal of Systems and Software*.

[8] Tao W., Chang D. (2019). News text classification based on an improved convolutional neural network. *Tehnicki vjesnik-Technical Gazette*.

[9] Arya A., Wijaya M. (2016). Modal sosial untuk kapasitas community governance (studi kasus perempuan pesisir kelurahan sulaa kota baubau). *JURNAL ILMU PEMERINTAHAN Kajian Ilmu Pemerintahan dan Politik Daerah*.

[10] Gaska K., Generowicz A., Zimoch I., Ciuła J., Iwanicka Z. (2017). A high-performance computing (h) based integrated multithreaded model predictive control (m) for water supply networks. *Architecture, Civil Engineering, Environment*.

[11] Thoman P., Dichev K., Heller T. (2018). A taxonomy of task-based parallel programming technologies for high-performance computing. *The Journal of Supercomputing*.

[12] Hut I., Jeftic B., Matija L., Cojbasic Z., Koruga D. (2019). Machine learning classification of cervical tissue liquid based cytology smear images by optomagnetic imaging spectroscopy. *Tehnicki vjesnik-Technical Gazette*.

[13] Noda I., Ito N., Izumi K., Mizuta H., Kamada T., Hattori H. (2018). Roadmap and research issues of multiagent social simulation using high-performance computing. *Journal of Computational Social Science*.

[14] Service R. F. (2016). China overtakes U.S. supercomputing lead. *Science*.

[15] Krasnopolsky B. I. (2018). Optimal Strategy for modelling turbulent flows with ensemble averaging on high performance computing systems. *Lobachevskii Journal of Mathematics*.

[16] Bouchard K. E., Aimone J. B., Chun M. (2018). International neuroscience initiatives through the lens of high-performance computing. *Computer*.

[17] John H. (2018). Blockchain technology. *Automotive recycling*.

[18] Sikorski J. J., Haughton J., Kraft M. (2017). Blockchain technology in the chemical industry: machine-to-machine electricity market. *Applied Energy*.

[19] Zhang Y., Wen J. (2017). The IoT electric business model: using blockchain technology for the internet of things. *Peer-to-Peer Networking and Applications*.

[20] Miraz M. H., Ali M. (2018). Applications of blockchain technology beyond c. *Annals of Emerging Technologies in Computing*.

[21] Yeoh P. (2017). Regulatory issues in blockchain technology. *Journal of Financial Regulation and Compliance*.

[22] Aptea S., Nikolai P. (2016). Will blockchain technology revolutionize excipient supply chain management?. *The Journal of Excipients and Food Chemicals*.

[23] Sun J., Yan J., Zhang K. (2016). Blockchain-based sharing services: what blockchain technology can contribute to smart cities. *Financial Innovation*.

[24] Beck R., Avital M., Rossi M., Thatcher J. B. (2017). Blockchain technology in business and information systems research. *Business & Information Systems Engineering*.

[25] Ittay E. (2017). Blockchain technology: transforming libertarian cryptocurrency dreams to finance and banking realities[J]. *Computer*.

[26] Engelhardt M. A. (2017). Hitching healthcare to the chain: an introduction to blockchain technology in the healthcare sector. *Technology Innovation Management Review*.

[27] Yuan Y., Zhou T., Zhou A. Y., Duan Y. C. (2017). Blockchain technology: from data intelligence to knowledge automation. *Zidonghua Xuebao/Acta Automatica Sinica*.

